# Design of Psychological Well-Being Education Environment Scheme Based on Deep Learning Theory

This article has been retracted.

**DOI:** 10.1155/2022/3460830

**Published:** 2022-09-01

**Authors:** Lingxia Guo

**Affiliations:** School of Marxism, North University of China, Taiyuan 030051, China

## Abstract

This paper discusses the structure of psychological well-being education programmes in higher education institutions based on an analysis of the connotation and characteristics of deep learning theory, as well as the background of today's talent training requirements, the psychological traits of contemporary students, and the practical requirements of the teaching reform of psychological well-being education courses in higher education institutions. A model for evaluating the psychological well-being of college students based on BPNN is presented in this paper, which also addresses the current severe shortage of full-time psychological counsellors. Additionally, the traditional BPNN is optimised by GA, and the resulting NN can better achieve the desired effect, demonstrating the viability of BPNN. It enables the psychological well-being of college students to be self-diagnosed online and significantly lessens the workload of psychological counselling institutions in higher education. According to the experimental findings, the optimised algorithm's accuracy can reach 92.47 percent, and it is considered to be reliable. This study not only offers a novel approach to nonlinear data processing, but also paves the way for variable screening in the presence of an ambiguous structure. Additionally, in a limited sense, it offers insightful research for psychological education in higher education institutions.

## 1. Introduction

Information technology has changed people's lifestyles, but it has also had an impact on their thinking and learning. This is especially true with the rise of the Internet and mobile devices, the development of “big data,” and artificial intelligence. The heavy responsibility of developing talent falls on institutions of higher learning, and the physical and mental health of college students directly affects the strength, stability, and success of the nation [1]. Implementing psychological well-being education in higher education institutions enriches their academic offerings, improves the quality of their teaching strategies, and elevates it to a crucial component of their daily instruction and management. However, in recent years, there has been a worrying decline in college students' psychological health, as well as an uptick in their psychological issues and the emergence of extreme events brought on by these issues [2]. As a result, both the students themselves and society as a whole have suffered serious consequences [3]. Problems with a student's psychological health have a direct impact on that student's overall quality as a college student as well as their general ability. It is necessary to sort out and talk about the pertinent theoretical issues of the psychological well-being education model in higher education institutions in light of this situation. The current classroom teaching reform has recently focused on deep learning, making it a hot topic. It has also come into teachers' focus to investigate and reform in-depth instructional design that is in line with in-depth learning. Deep learning [4, 5] is defined as learning in which students pay close attention to the meaning and importance of the material they are learning. Deep learning entails continuously creating new schemas while revising existing ones. After many years of study, the theory of deep learning has reached the point of steady advancement and practical application. To enhance students' capacity for learning, all disciplines are attempting to investigate the use of deep learning mode in instruction.

It is impossible to attain the objective of all-around development without students having a healthy personality, healthy psychology, and harmonious interpersonal relationships. As a result, in order to strengthen psychological well-being education, higher education institutions are needed [6]. The work of teaching college students about their psychological well-being is modern and relevant. New and better ways and means are required as a result of societal development. A type of individualised, meaningful exploration and discovery learning and deep learning is used in the field of education. To put it another way, learners build a new knowledge framework to enhance their own knowledge system by considering and critiquing new knowledge based on the original knowledge framework, integrating the old and the new, transferring, and verifying it [7]. A learning plan, which is an essential supporting tool in the teaching process, aims to develop students' capacity for independent learning and direct students in structuring their knowledge through questions, in line with the workings of deep learning. In the course of learning, deep learning places more emphasis on the path taken by students and their psychological state [8]. In addition to being a new requirement for teaching and learning in the modern era, deep learning is the benchmark for students' autonomous learning effects. It supports both the thorough development of curriculum teaching reform and the promotion of students' comprehensive mastery of what they have learned. From the standpoint of educational objectives, Bloom's classification of educational goals cannot be separated from the development of learning objectives in lesson plans, whereas deep learning refers specifically to Bloom's highest level of cognitive objective classification system, the level of advanced cognitive skills [9]. Fundamentally connected are the two. Instead of the traditional external indoctrination and passive acceptance of shallow learning, it can be used to apply the knowledge and skills learned to solving practical problems. This paper examines the design of a programme for teaching psychological well-being based on the deep learning theory. The innovations of this paper are as follows:

1. Aiming at the serious shortage of full-time psychological counsellors at present, this paper puts forward an evaluation model of college students' psychological well-being based on BPNN (back propagation neural network). It can realize online self-diagnosis of college students' psychological well-being and greatly reduce the work pressure of psychological counselling institutions in institution of higher learning.
2. In this paper, GA (genetic algorithm) is used to optimize the traditional BPNN, which is easy to fall into the local minimum, slow in convergence, and uncertain in generalization ability of the network. The optimized NN (neural network) can achieve the expected effect better, which shows the feasibility of this method.

This paper aims to study the design of psychological well-being education scheme. The article consists of five sections, with the specific structure as follows.

## 2. Related Work

According to the characteristics of students' physical and mental development, Primack et al., with the help of experiential teaching activities, used painting, four-square grid, group counselling, and other methods to teach in the psychological well-being education classroom to promote students' in-depth learning [10]. Hartley pointed out that adhering to the in-depth learning-oriented classroom teaching will further promote the reform and development of college psychological well-being education teaching and comprehensively improve the quality of classroom teaching. It helps to consolidate the foundation of college students' psychological well-being knowledge and improve their psychological quality and psychological well-being literacy [11]. Markoulakis and Kirsh pointed out that paying attention to the psychological development of college students, strengthening the work of psychological well-being education, and truly training them to become socialist builders with both political integrity and physical and psychological well-being are a new topic facing higher education [12]. Combining NN and psychological well-being education research, Albright and Hurd proposed a psychological well-being assessment model based on BPNN [13]. Zhang and Du expounded the necessity of implementing psychological well-being education in institution of higher learning; analyzed the requirements of social development, the requirements of school education goals, and the requirements of students' personality development; and pointed out the urgency of implementing psychological well-being education in institution of higher learning [14]. In order to further optimize the model recognition effect, Downs et al. proposed a psychological well-being problem recognition algorithm based on the DeepPsy model [15]. Combining with the current situation and characteristics of the student group, Rosen et al. expanded the evaluation factors by analyzing the reasons that affect the students' psychological well-being; they collected the corresponding data and used the NN model to predict and analyze the students' psychological well-being status [16]. Levecque et al. revealed the main countermeasures and approaches for college students' psychological well-being education from the aspects of higher education authorities, university management, teachers, campus cultural environment, and the relationship between psychological well-being education and ideological and political education [17]. Labrie et al. pointed out that the enlightenment of positive psychology to psychological well-being education is reflected in the integration of goals, the improvement of health level, the cultivation of healthy personality, and the improvement of a harmonious educational environment [18]. Davies et al. pointed out that psychological well-being education is faced with insufficient understanding, problems in the implementation process, deficiencies in curriculum construction, and teacher team construction [19]. Although scholars have studied and explored the psychological well-being education model in institution of higher learning from different perspectives, they have proposed a variety of psychological well-being education models and applied them to practical work. However, many models have their own problems.

The psychological well-being of students is assessed in this paper using NN theory [20] and technology, and a new model for assessing and categorising psychological well-being is developed. In this study, the distinctive psychological well-being indicators are isolated from the challenging test items to create a specific set. Then, the key influencing variables in the assessment of psychological well-being are chosen as input vectors, and the BPNN model is used to assess the psychological well-being status. The traditional BPNN is optimised using GA in order to address the issues that it has with slow convergence, a tendency to fall into local minima, and an unreliable generalisation capability. In order to obtain the output results, training samples are provided. The output results are then analyzed, and the results of the various algorithms are contrasted. According to the research, the method suggested in this paper not only increases the mathematical model's accuracy but also gives the impression of being more straightforward, efficient, and scientific.

## 3. Methodology

### 3.1. Overview of Psychological Well-Being Education

The creation of psychological well-being education was done so as to meet the demands of both social development and the development of personal psychological well-being. The goal of psychological well-being education is to address the developmental issues that ordinary people face, such as career planning and personality enhancement, while also addressing students who may have psychological barriers or issues. According to the concept of big education, psychological well-being instruction in higher education institutions counts as educational activity. This includes psychological counselling, psychological consultation, and psychological treatment, in addition to the teaching of courses on psychological well-being and the promotion of this knowledge. Psychological well-being education has a richer connotation than psychological counselling and counselling, at least in terms of connotation. Higher education institutions bear a heavy burden of nurturing talent in the twenty-first century, and the success of individuals as well as the strength and stability of the country is directly correlated with the physical and mental health of college students. Therefore, it is important for college students' overall development to provide moral guidance and mental enlightenment, enhance their personality systems, and encourage these processes. This paper asserts that psychological well-being education is a type of educational activity in which educators use the theories and techniques of psychology and related disciplines to aid students in solving their psychological problems as they grow and to promote the improvement of all students' psychological quality and the healthy development of their mental functions throughout the educational process. The approach to teaching psychological well-being in higher education institutions is a symbol of how this subject has evolved from disorder to order, from the level of experience to the level of science. It is the result of practice, and at the same time, it has a significant role in directing the delivery of psychological well-being education in higher education institutions. Educational objectives, educational contents, educational approaches, evaluation, and management mechanisms are all components of the model for teaching psychological well-being in higher education institutions. Numerous psychological issues among college students have unquestionably increased as a result of the current social life rhythm's acceleration and the competition's escalating ferocity, and the government, society, universities, and individual students have all begun to pay increasing attention to these issues. This work's foundation and assurance of a healthy and thorough development are a full understanding of the necessity and significance of educating college students about their psychological well-being.  Figure 1 shows the current situation of college students' psychological well-being content.

Psychological well-being education is a purposeful, planned, and organized process of influencing students' mental quality. In order to ensure the smooth progress of this process, we must construct a practical general goal of psychological quality education in institution of higher learning. The formulation of this goal should take into account not only the current social development's need for talents, but also the characteristics of college students' physical and mental development. It is of great significance to scientifically establish the target system of psychological well-being education in institution of higher learning for constructing the model of psychological well-being education in institution of higher learning. If the quality of psychological well-being is a stable psychological trait, then psychological well-being is a complete state of psychological well-being that is full of vitality, can effectively exert one's potential to adapt to the environment, and has positive inner experience [21]. The general goal of psychological well-being education in institution of higher learning is to improve the overall psychological quality of college students and make their personality harmonious; improve its social adaptability; enhance college students' self-psychological education ability; solve all kinds of developmental problems faced by college students in their development; and prevent and reduce mental illness. The content of psychological well-being education is the embodiment of the goal of psychological well-being education, which is directly related to the realization of the goal of psychological well-being education, and it is an important link.

Psychological education has the following principles: (1) systematic principle, (2) educational principle, (3) principle of subjectivity, (4) principle of totality, (5) principle of difference, and (6) scientific principle. In the view of positive psychology, college students' psychological well-being education is student-centered and starting point. The selection of teaching contents and the application of teaching methods should fully respect the law of college students' physical and mental development and their growth needs, so as to give full play to their initiative. Psychological well-being education in institution of higher learning is a kind of quality education for all college students and a systematic project. It should be incorporated into the overall system of school education to give full play to the overall benefits of school education. The demand for talents in the new era requires young college students to develop in an all-round way and have a high level of comprehensive quality. We should not only be physically and mentally healthy, but also have a strong physique and strong psychological quality. We should also have both ability and political integrity, solid professional knowledge, and good ideological and moral quality to meet the needs of social development. To sum up, the main contents of college students' psychological well-being education should include the following aspects: (1) education of sound personality, (2) interpersonal harmony education, (3) actively adapting to education, and (4) independent psychological education. College students' psychological well-being education is a complex systematic project, and it needs effective ways to implement it, so as to effectively accomplish the task of psychological well-being education and cultivate talents with good psychological quality. Strengthening college students' psychological well-being education is the internal need to improve college students' psychological well-being. At the same time, it is also an urgent requirement to improve the psychological well-being education in institution of higher learning.

### 3.2. Design Strategy of Educational Scheme Based on Deep Learning

Due to the late start of psychological well-being education in institution of higher learning, and the influence of many factors, such as ideological understanding, working conditions, and teachers' level, the current development of psychological well-being education in institution of higher learning is very unbalanced, and there are still many inadequacies in the working system, ways, and methods. All teachers are necessary for the development of psychological well-being education, and the calibre of the teachers affects the calibre of the education. Teachers are crucial in bridging the gap between classrooms and students, and they are also the main conduits through which psychological well-being education knowledge is disseminated. Presently, classroom instruction, psychological consultation rooms, lectures, etc. are the primary methods used by teachers to disseminate knowledge about psychological well-being education. This type of educational approach is dull, lacks teacher-student interaction, and yields a teaching outcome that is only half as effective as it could be. It is unable to change to meet the demands of students and the advancement of society. Therefore, we should muddy up the concepts of pure psychology and physiology and emphasise the life and practicality of teaching content in order to combat the adult, systematic, and theoretical tendency in textbooks. In addition, teachers and students should focus on improving communication, inspiring students to recognise their own excellent qualities, and preventing psychological issues. Schools should promote psychological knowledge more widely and raise teachers' awareness of the importance of psychological well-being education. At the same time, psychological well-being education should adopt a treatment-assisted, education-focused approach to its delivery. In psychological well-being education classes, teachers should pay attention to student differences and encourage in-depth study to varying degrees; at the same time, we should pay attention to the autonomy of student growth and encourage the autonomous occurrence of deep learning.

Education about psychological well-being is a crucial component of education and is inextricably linked to classroom instruction and learning. The improvement of teachers' professionalism, not only in psychological well-being courses but also in other professional courses, and the relationship between teachers and students are the development directions for psychological well-being education. College instructors should take the best parts of psychological well-being education, apply them to their own work, and use them for “self.” In order for all educational work to pay more attention to students' most fundamental and general psychological needs while also paying attention to the requirements of society on individual politics, ideologies, and behaviour norms, it is necessary to take the development of students' psychological qualities as one of their own goals and contents. Real life and education are inseparable. By putting students in situations that are similar to those in their real lives when creating learning plans, teachers can guide students' values in a welcoming and inclusive learning environment, contributing to keeping things quiet. Indirect experience, which gives students the internal logic and knowledge structure to understand knowledge and can encourage students' divergent thinking, is another method by which students can learn deeply. Additionally, we need to create a teaching methodology that aims to raise the psychological standards of college students in order to implement the psychological well-being education. The teaching system should take psychological well-being education as the main line, make it closely integrated with other subject courses and activity courses, promote each other, coordinate and cooperate with each other, and infiltrate psychological well-being education into all subject teaching. This will not only help to improve college students' psychological quality and psychological well-being education level, but also help to improve the present situation of various subjects' teaching and achieve a win-win situation. Learning objectives can help learners transform their learning from shallow cognition and memory to deep thinking, reflection, and judgment and from focusing on the concept of learning to focusing on the process of learning. Deep learning aims to help students improve their ability to understand and solve problems in different situations.

Teachers should follow the “developmental” teaching concept and the principle of comprehensive and all-round development teaching before creating a deep learning classroom for psychological well-being education in a higher education institution. This will help teachers to encourage students' significant development in cognition, emotion, skills, morality, and psychological quality through classroom instruction. College students who want to learn about psychological well-being should focus on both how to fully utilise their advantages as students as well as how to pay attention to mental illnesses. In addition to treating illnesses, it emphasises the role that educational activities play in fostering students' ability development. Openness, acceptance, and tolerance are qualities of psychological well-being education courses. The psychological well-being education course for college students should be based on upholding the proper values. The development of thought is essential to the process of designing a learning plan. The development of higher-order thinking is one of the learning goals that are outlined in the learning plans. Another goal is to create a reasonable and perfect knowledge framework that will enable students to think creatively. A third goal is to foster cognitive conflict so that students' thinking can grow and become more in-depth. To summarise, institutions of higher education should improve the leadership and management of psychological well-being education, actively promote the growth of psychological well-being education in institutions of higher education, and assist in resolving challenges and issues at work.

### 3.3. NN-Based Evaluation Model of College Students' Psychological Well-Being

Evaluations of mental health and the identification of psychological issues are essentially nonlinear classification or pattern recognition issues. Each person's psychological state is a multidimensional information system with the basic properties of multivariable, multilevel, and strong coupling. There are also complex nonlinear interactions between the system's various components. Thus, it is challenging to formulate it in terms of conventional mathematical techniques. In this study, the psychological well-being evaluation model for college students is modeled using the NN algorithm. In order to simulate this abstract process through computer programmes, NN will take some fundamental characteristics of the nervous system from which the biological brain responds to stimuli. By using the neuron mathematical model and Hebb learning rules to learn a large number of examples, NN supports decision-making by identifying new examples. Following are some benefits of NN: (1) It is capable of approximating every complex nonlinear relationship in full. (2) It is highly resilient and fault tolerant. (3) A distributed parallel processing approach is used, allowing for the quick execution of a significant number of operations. (4) Develop your ability to adapt to new or hazy systems. (5) Possess the capacity to work with both quantitative and qualitative knowledge. Through a simulation of the brain's response mechanism, in which information is sensed from the receptor and the effector reacts to the sensed information, NN is the process of processing and analyzing the received information and providing the processing result to the effector to issue some sort of command. NN is a method that combines qualitative and quantitative techniques to aid in decision-making. In contrast to the quantitative approach, which uses neurons, the qualitative approach focuses on knowledge-based reasoning. Calculation is a key component of the information processing process. The structure of NN is shown in Figure 2.

The BPNN model is a hierarchical network with three or more layers in which all neurons in the adjacent upper and lower layers are connected; that is, each neuron in the lower layer is connected with each neuron in the upper layer, but there is no connection between neurons in each layer. Its basic tenet is that, by continuously learning from sample data, NN uses adaptive ability to adjust each neuron's error threshold, causing the error function of the network output and the anticipated output to be adjusted in the direction of gradient decline. In addition to input and output nodes, BPNN also has one or more hidden nodes. It is currently the NN model that is used the most.  Figure 3 depicts the overall architecture of the algorithm used to evaluate issues with students' psychological well-being based on data from multiple sources.

In GA, the individual's viability is described by the individual's fitness, which is the degree of conformity with the problem objectives. The optimal solution is to find the individual with the largest fitness value through the iterative process of the algorithm. The fitness functions mainly include the following: if the objective function is the minimum problem, then

(1) $$\begin{array}{c} \text{Fit}\left(X\right)=\left\{\begin{array}{cc} C_{\max}-f\left(X\right), & \text{if }f\left(X\right)<C_{\max},\\ 0, & \text{else}, \end{array}\right. \end{array}$$

and if the objective function is a maximum problem, then

(2) $$\begin{array}{c} \text{Fit}\left(X\right)=\left\{\begin{array}{cc} C_{\min}+f\left(X\right), & \text{if }f\left(X\right)+C_{\max}>0,\\ 0, & \text{else,} \end{array}\right. \end{array}$$

where *C*_min_ is a given smaller number and *C*_max_ is a given larger number. According to the specific problem, choose the appropriate fitness function. The higher the fitness, the greater the probability of being selected; that is, the relationship between the probability *P*_*i*_ of the individual *i* being selected and the fitness *F*_*i*_ is

(3) $$\begin{array}{c} P_{i}=\frac{F_{i}}{\sum_{i=1}^{M}F_{i}}\;i=1,2,3,\ldots ,M. \end{array}$$

For an ordinary set *A*, any element *x* is in the space, either *x* ∈ *A* or *x* ∉ *A*. The two must be one or the other. This feature can be represented by a function as

(4) $$\begin{array}{c} A\left(x\right)=\left\{\begin{array}{cc} 1, & x\in A,\\ 0, & x\notin A. \end{array}\right.. \end{array}$$

Among them, *A*(*x*) is the characteristic function of the set *A*. The feature function is generalized to fuzzy sets, and only two values of 0 and 1 are taken in the ordinary set to generalize to the [0, 1] interval of the fuzzy set. Build a judging set:

(5) $$\begin{array}{c} V=\left\{v_{1},v_{2},v_{3},\ldots ,v_{n}\right\}. \end{array}$$

Establish a single-factor judgment; that is, establish a fuzzy mapping from *U* to *F*(*V*):

(6) $$\begin{array}{c} f:U⟶F\left(V\right),\forall u_{i}\in U,\\ u_{i}|⟶f\left(u_{i}\right)=\frac{r_{i1}}{v_{1}}+\frac{r_{i2}}{v_{2}}+\cdots +\frac{r_{im}}{v_{m}},\\ 0\leq r_{ij}\leq 1\;1\leq i\leq n\;1\leq j\leq m. \end{array}$$

The fuzzy relationship can be induced by *f*, and the fuzzy matrix can be obtained:

(7) $$\begin{array}{c} R=\left[\begin{array}{cccc} r_{11} & r_{12} & \ldots & r_{1m}\\ r_{21} & r_{22} & \ldots & r_{2m}\\ \ldots & \ldots & \ldots & \ldots \\ r_{n1} & r_{n2} & \ldots & r_{nm} \end{array}\right]. \end{array}$$

Among them, *R* is a single-factor evaluation matrix, so (*U*, *V*, *R*) constitutes a comprehensive evaluation model.

This paper obtains four data sources during the data acquisition and preprocessing stages: network log, access control data, achievement data, and consumption data. This paper uses four data sources to extract the related features of students' online behaviour and abnormal consumption scores during the feature extraction stage. The most effective classifier is chosen from five widely used classification algorithms during the model training and recognition stage. With 6 neurons in the input layer, 5 neurons in the output layer, and 7 neurons in the hidden layer, the sample is built as a NN. The input and output of each neuron in a feed-forward network called a perceptron model are discrete values. Each neuron's output is determined by the threshold function after its input is weighted and summed. Its output can be expressed as follows if the weighted sum of the inputs is *y*, which is also the NN's output:

(8) $$\begin{array}{c} y=f\left(\sum_{j=1}^{n}w_{j}u_{j}-\theta \right)=f\left(\sum_{j=0}^{n}w_{j}u_{j}\right),\\ w_{0}=-\theta \;u_{0}=0, \end{array}$$

where *u*_*j*_ is the *j* th input of the perceptron. The model goals are

(9) $$\begin{array}{c} E=\frac{1}{2}\sum_{p=1}^{P}\sum_{k=1}^{L}{\left(T_{k}^{p}-O_{k}^{p}\right)}^{2}. \end{array}$$

The trained NN can approximate the ideal output by new input; that is, the error between the actual output and the ideal output is the smallest.

## 4. Result Analysis and Discussion

The connection weights and thresholds of each NN factor are given the best possible solution, and NN then modifies the weights and thresholds. This is known as applying GA to NN. It is possible that the weight threshold that the GA algorithm optimises for will be closer to the value needed by the network. In general, NN employs the equal Hamming distance coding method for both its input and output. Input from the network is the factor score of the index, and the network outputs three measurement results—healthy, slightly unhealthy, and unhealthy—that are each coded as 100, 010, and 001, respectively. The construction of the NN for evaluating the psychological well-being of college students uses six types of common mental disorders among students as training data.  Table 1 shows the training set of college students' psychological well-being identification.

The model requires real data sets, which are typically split into training sets and testing sets, for the training and testing phases. The sample data are divided into two parts at random, one of which is used as training samples to train the network and the other as testing samples to test the trained network and then determine whether it satisfies the requirements. The momentum term added in the enhanced network is initially given the value 0.7, and the network's learning rate is set to 0.51 per second. The network will go through 4000 training cycles, with a training error expectation of 0.00001. The input and output sample data are similar to those of the BPNN, where the network adopts a three-layer structure, allowing for a comparison between the simulation results of the two types of neural networks.  Figure 4 shows the training of different networks.

The convergence speed of BPNN is evidently faster than that of CNN during network training, and both the training results and network output results exhibit good stability. Once you have the model service prototype, convert it into C# language source code and save it in the file proxyclass.cs. The programme that will use this class should include this file in the DSS client project and make use of its namespace. To ascertain whether the prediction model can fulfil the anticipated prediction purpose, the model is simulated and tested. The trained model is more likely to favour the dataset with more samples because the data is unbalanced. We use time splitting to increase the number of positive samples in order to get around this issue and balance the positive and negative sample counts in the training set. The accuracy of the algorithm is displayed in Figure 5.

With the support of WebServices model service and database system, it is easier to develop the client application of psychological barrier identification decision support system. After the NN training, input the default conditions for the samples. By calculating the error between the actual output and the ideal output, the output error of each layer of neurons is adjusted from the output layer of the network; that is, the weight threshold of neurons is adjusted according to the gradient descent method, and the actual output obtained by the network can be basically close to the ideal output through continuous back propagation. The stability results of the system are shown in Figure 6.

Run the client program to get the reasoning result report. The report includes the following contents: (1) input parameters after text to value conversion; (2) calculate output value of NN; (3) the final conclusion is based on the output value. After the training, test with the test sample data. See Table 2 for the results.

Because of the generalization function of NN, the trained network can also give appropriate output for inputs that are not in the sample set. Therefore, fuzzy mathematics can be used to transform a person's qualitative evaluation of routine performance and personality into quantitative evaluation-membership degree. Then it can be used as input data to diagnose which level of a person's mental state, and then it can give more scientific suggestions for diagnosis and treatment. See Figure 7 for the comparison result between the expected value of the sample and the actual output value of the model.

It can be seen from all the data that the modeling of psychological well-being based on BPNN has good accuracy and adaptability, the error of the modeling results is small, the fitting is good, and the modeling results are obviously better than those of CNN. In this paper, through the effective combination of the two algorithms, the advantages of the two algorithms are complementary. The optimised NN not only improves the learning speed, but also greatly improves the approximation ability and generalization ability of the whole network during the training process. Experiments show that the accuracy of this algorithm can reach 92.47%, and the algorithm has certain reliability.

## 5. Conclusions

Psychological well-being education is a crucial component of a curriculum meant to develop students' personalities and souls. It also helps to develop students' potential. For psychological well-being education among college students to be effective, many fundamental changes must be made. Higher-order thinking skills can be developed in students by combining in-depth study with a learning plan and instruction. This essay examines how deep learning theory can be used to create effective lesson plans in the context of a psychological well-being education classroom. There is no correlation between these factors, however, and the research on issues with psychological well-being is very complex. The main problem now is how to solve this nonlinear relationship. This study uses the NN algorithm to model the psychological well-being evaluation model of college students due to the intricate relationship between different influencing factors and their mental state. The traditional BPNN is easy to fall into the local minimum in this paper, the convergence speed is slow, the network's ability to generalize is unsure, and so on. The conventional BPNN is enhanced by GA. This method is feasible because the optimised NN can produce the desired effect more effectively. According to the experimental findings, the optimised algorithm's accuracy can reach 92.47 percent, and it is considered to be reliable. This study offers some useful research for higher education institutions' psychological curricula. The severity of students' psychological well-being issues cannot be predicted using this method, though. I want to be able to gauge how serious the issues affecting students' psychological well-being will be in my future work.

## Figures and Tables

**Figure 1:** Status quo of college students' psychological well-being content.

**Figure 2:** NN structure.

**Figure 3:** The overall framework of the evaluation algorithm.

**Figure 4:** Training situation of different networks.

**Figure 5:** Accuracy performance of the algorithm.

**Figure 6:** Stability result test of the system.

**Figure 7:** Errors between different expected outputs of the network and the actual output values of the model.

**Table 1:** Training set of college students' psychological well-being identification.

Symptom	Depression	Obsessive-compulsive disorder	Anxiety disorders	Phobia	Suspected illness	Schizophrenia
Somatic symptoms	Loss of appetite		Muscular tension			

Behavioral symptoms	Decreased speech action	Obsessive behaviour		Avoidance behaviour	Repeated visits	Delusion

Emotional symptoms	Serious inferiority complex	Obsessional thoughts	Worried, nervous	Horrible emotion	Suspicion of illness	

Sleep symptoms	Severe insomnia	Poor sleep	Difficult to sleep	Poor sleep		

Interpersonal symptoms	Self-closing					Do not trust others

**Table 2:** Test results of different networks.

Number	Expected output	BPNN output	CNN output
1	1, 0, 0	0.8737, −0.0031, 0.0068	0.8960, −0.0018, −0.0096
2	1, 0, 0	0.7998, −1.6273, 3.4451	0.8378, 0.0369, 0.0361
3	1, 0, 0	0.8665, −0.0004, 0.0008	0.8730, 0.0039, 0.0061
4	1, 0, 0.	0.8826, 0.0039, −0.0083	0.8550, 0.0084, 0.0073
5	1, 0, 0	0.9511, 0.0001, −0.0003	0.9349, −0.0184, −0.0134
6	1, 0, 0	0.9407, 8.9052, −0.0001	0.9229, −0.0049, −0.0134
7	1, 0, 0	0.92503, −0.00059907, 0.0012	0.9163, −0.0086, −0.0096
8	0, 1, 0	−8.7254, 0.9999, 2.2282	−0.0013, 0.9993, 0.0063
9	0, 1, 0	0.0004, 1, −0.0001	−0.0002, 0.9982, −0.0007
10	0, 1, 0	−1.1252, 1, 2.8733	−0.0075, 1.0002, 0.0052

## Data Availability

The data used to support the findings of this study are available from the author upon request.
